RETRACTED

# Effect of Dexmedetomidine on Postoperative Lung Injury during One-Lung Ventilation in Thoracoscopic Surgery

**DOI:** 10.1155/2020/4976205

**Published:** 2020-10-05

**Authors:** Jun Meng, Qin Lv, Jiaxiang Yao, Siyu Wang, Kun Yang

**Affiliations:** ^1^Department of Cardiovascular Surgery, First Affiliated Hospital of Kunming Medical University, Kunming 650032, China; ^2^Department of Anaesthesiology, First Affiliated Hospital of Kunming Medical University, Kunming 650032, China

## Abstract

**Objective:**

To investigate the effect of dexmedetomidine on postoperative lung injury in patients undergoing thoracoscopic surgery.

**Methods:**

From March 2019 to October 2019, 40 patients were randomly divided into two groups: dexmedetomidine group (group D) and control group (group C). Except recording the general condition of the patients in both groups preoperatively and intraoperatively, the oxygenation index (OI) and alveolar-arterial oxygen partial pressure difference (A-aDO_2_) were monitored at admission (T0), immediately after one-lung ventilation (T1), 0.5 h after one-lung ventilation (T2), and 15 minutes after inhaling air before leaving the room (T3). The content of IL-8 in arterial blood was measured by enzyme-linked immunosorbent assay (ELISA) at T0 and T2, and the expression of AQP1 protein in isolated lung tissue was measured by immunohistochemistry and Western blot. The incidence of postoperative pulmonary complications (atelectasis, pneumonia, and acute respiratory distress syndrome) was used as the index of lung injury.

**Results:**

There was no significant difference in the general condition before and during operation between the two groups. There was no significant difference in arterial blood IL-8 content between the two groups at the T0 time point, but the arterial blood IL-8 content at the T2 time point was significantly higher than that at the T0 time point, especially in group C. The results of immunohistochemistry and Western blot showed that the expression level of AQP1 protein in the isolated lung tissue of group D was significantly higher than that of group C (*P* < 0 05). At T3, the OI of group D was significantly higher than that of group C, and the A-aDO_2_ of group D was significantly lower than that of group C (*P* < 0.05). There was no significant difference in the incidence of postoperative PPCs between the two groups.

**Conclusion:**

Dexmedetomidine can reduce the level of plasma IL-8 and upregulate the expression of AQP1 in the lung tissue of patients undergoing thoracoscopic surgery under one-lung ventilation, but it has no significant effect on the incidence of postoperative PPCs. Dexmedetomidine can be safely used in thoracoscopic surgery and has a certain protective effect on lung injury.

RETRACTED

## 1. Introduction

Acute lung injury (ALI) has become the main cause of death after thoracic surgery and has the characteristics of high incidence (2-5%) and mortality (>25%). In addition to the causes of the operation itself, intraoperative mechanical ventilation (MV) is considered to be one of the important causes of ALI [1, 2]. At present, it is considered to be caused by the release of inflammatory mediators caused by nociceptive ventilation modes (high tidal volume, high peak inspiratory pressure, high inhaled oxygen concentration, etc.). Especially in one-lung ventilation (OLV), the body relies on one side of the lung for oxygenation, resulting in an increase in intrapulmonary anatomical shunt, which can easily to cause hypoxia and lung injury [3]. Human and animal experimental studies have shown that even if protective ventilation strategies are adopted (low tidal volume, low peak inspiratory pressure, reduced inhaled oxygen concentration, etc.), it cannot completely prevent the production of inflammatory mediators in lung tissue and the occurrence of lung injury [4–7].

ALI is a pathological process characterized by increased pulmonary permeability and lung inflammation. IL-8 is a sensitive index of airway inflammation [8]. IL-8 can activate and chemotactic neutrophils and cause airway neutrophils to gather and activate, thus promoting inflammation and aggravating airway inflammation. IL-8 plays an important role in the pathogenesis of lung injury and pulmonary interstitial diseases [9], and its concentration level can reflect the degree of lung injury to a certain extent. Aquaporin-1 (AQP1) is a kind of aquaporin, which can selectively and actively transport water. AQP1 is mainly distributed in the lung tissue. When its expression or activity decreases, the liquid in the interstitial lung will clear up obstacles, which will lead to a large amount of liquid accumulation between the alveoli, interstitial lung, and capillaries and cause or aggravate pulmonary edema [10], which plays a vital role in the occurrence and development of ALI.

Dexmedetomidine is a new type of agonist of *α*-2 adrenergic receptor with high selectivity, which can inhibit the release of norepinephrine after being stimulated by drugs. Dexmedetomidine has central antisympathetic properties, thus playing a sedative, analgesic, and anxiolytic role, and has been widely used in clinical anesthesia. Many studies have shown that dexmedetomidine can alleviate inflammatory reaction. Therefore, we put forward the scientific hypothesis that dexmedetomidine can exert lung protection by inhibiting the production of IL8 and upregulating the expression level of AQP.

RETRACTED

In this study, the level of serum IL-8 and the expression of AQP1 in the lung tissue of surgical patients were detected, and the incidence of postoperative pulmonary complications (atelectasis, pneumonia, and acute respiratory distress syndrome) was taken as the judgment index of lung injury, so as to explore the effect of dexmedetomidine on postoperative lung injury of patients undergoing thoracoscopic surgery under one-lung ventilation.

## 2. Materials and Methods

### 2.1. Research Objects

This experiment was approved by the Ethics Committee of the First Affiliated Hospital of Kunming Medical University (Lunshen L No. 37, 2019), with the consent of the patients and their families and signed informed consent forms. A total of 40 patients who underwent elective thoracoscopic lobectomy (TL) in the First Affiliated Hospital of Kunming Medical University from March 2019 to October 2019 were selected. All patients were ASA I-II, aged 30-70 years, and their body mass index was 18-30 kg/m^2^. According to the eighth edition of staging standard of International Association for Lung Cancer Research (IASLC), all the selected lung cancer patients were in stage IA. They were randomly divided into dexmedetomidine group (group D) and control group (group C), 20/group.

### 2.2. Exclusion Criteria

The exclusion criteria are as follows: serious infectious diseases before operation, with high infection index (C-reactive protein > 50 mg/L); preoperative sinus bradycardia or atrioventricular block; those who have a history of chemotherapy, radiation exposure, thoracic organ surgery before operation, and have stopped smoking for less than one week; severe hypertension and untreated before operation, history of diabetes and severe hepatic and renal insufficiency; suffering from severe COPD or extremely severe reduction of lung function before operation (FEV1% < 40; FVC% < 60; DLCO% < 60); anemia before operation (HB < 90 g/L); airway pressure > 30 mmHg or SPO_2_ < 90% during one-lung ventilation (OLV) during operation; patients with intraoperative blood loss > 300 mL, transfusion > 2500 mL, and intraoperative blood transfusion; and the operation time was less than 1 hour or more than 4 hours.

### 2.3. Anesthesia Management

Routine prohibition of drinking and fasting were executed before operation. The operation and anesthesia of all patients were performed by the same group of surgeons and the same group of anesthesiologists. The whole process of the experiment was double-blind. After entering the operating room, noninvasive blood pressure (NBP), heart rate (HR), finger pulse oxygen saturation (SPO_2_), and electrocardiogram (ECG) were routinely monitored to open the venous pathway of the upper limb. Radial artery catheterization was performed under local anesthesia, and invasive arterial blood pressure was monitored. Anesthesia induction and maintenance drugs in the two groups were the same: anesthesia induction: fentanyl 3 *μ*g/kg, propofol 2 mg/kg, and vecuronium 0.1 mg/kg intravenous injection; anesthesia maintenance: intravenous infusion of propofol 6-8 mg/(kg h) and remifentanil 0.15-0.25 *μ*g/(kg min) and intermittent injection of vecuronium to maintain satisfactory muscle relaxation. The BIS value during the maintenance operation was in the range of 40-60. In group D, right medetomidine 1 *μ*g/kg (finished within 10 minutes) was injected intravenously before induction; then, 0.5 *μ*g/(kg h) was injected intravenously until 10 minutes before the end of operation, and group C was injected with the same amount of normal saline. After anesthesia induction, all patients were intubated with double-lumen endotracheal tube (male 37F; female 35F Covidien Llc). The position of the catheter was adjusted under a fiber-optic bronchoscope and connected to the anesthesia machine (GE, Datex-Ohmeda Inc.) for volume-controlled mechanical ventilation. The mechanical ventilation parameter setting is as follows: [11]: tidal volume (VT) 6-8 mL/kg, frequency (f) 12-15 times/min, PEEP 5 cmH_2_O, *I* : *E* = 1 : 2, FIO_2_ = 1.0, and PETCO_2_ maintained in the range of 35-45 mmHg. Patients in both groups were treated with the same intraoperative fluid replacement regimen: compensatory dilatation volume, cumulative loss, physiological requirement, intraoperative blood loss, and loss of the third space, in which the compensatory dilatation capacity was 5 mL/kg, and the infusion was completed before anesthesia induction; cumulative loss = physiological requirement × fasting time. Physiological requirements were as follows: the first 10 kg infusion liquid 4 mL/kg, the second 10 kg infusion fluid increased by 2 mL/1 kg, infusion fluid increased by 1 mL/kg upon 20 kg, half of the liquid to supplement the first hour of infusion, the rest of the fluid in the next 2-hour infusion, and the third space loss according to 4 mL/(kg h) infusion. The compound electrolyte and hydroxyethyl starch were used for intraoperative infusion, and the sodium chloride injection was continuously infused at 1 : 1 according to the crystal-binder ratio. The intraoperative blood pressure was maintained at ±20% of the changes in preoperative resting blood pressure 60-100 times/minute; when hypotension or bradycardia occurred during the operation, the corresponding cardiovascular active drugs were given, respectively. Parecoxib, a no-steroidal anti-inflammatory and analgesic drug, 40 mg/kg was given half an hour before the end of the operation, and postoperative PCIA was used for analgesia, fentanyl 20 *μ*g/kg, 10 *μ*g/mL, continuous pump for 48 h.

RETRACTED

### 2.4. Observation Index

The general preoperative conditions (age, height, body mass index, operation site, and operation method) and intraoperative conditions (blood loss, infusion volume, operation time, one-lung ventilation time, bradycardia, and anesthetic dosage) were recorded in the two groups. The heart rate (HR), mean arterial pressure (MAP), oxygenation index (OI), and alveolar-arterial oxygen partial pressure difference (A-aDO_2_) were measured before admission (T0), immediately after OLV (T1), OLV 0.5 h (T2), and 15 minutes after breathing air before leaving the operating room (T3). The frequency of intraoperative hypotension (MAP < 60 mmHg) and bradycardia (HR < 50/min) was recorded. The content of IL-8 in arterial blood was measured by enzyme-linked immunosorbent assay (ELISA) at T0 and T2 time points. The expression of AQP1 protein in the isolated lung tissue was detected by immunohistochemistry and Western blot. The incidence of postoperative pulmonary complications (PPCs) was observed and recorded.

### 2.5. Evaluation Index of Pulmonary Inflammatory Reaction

Serum IL-8 concentration was used as an index to reflect the inflammatory reaction of the lung. Enzyme-linked immunosorbent assay (ELISA) was used to measure the serum IL-8 concentration at T0 and T2 time points.

### 2.6. Evaluation Index of Pulmonary Interstitial Water Permeability

The expression level of AQP1 in the isolated lung tissue was used as an evaluation index of interstitial water permeability of the lung.

#### 2.6.1. Immunohistochemical Staining and Protein Average Optical Density Analysis

1 × 1 × 1 cm^3^ normal lung tissue (more than 3 cm away from tumor and nontumor tissues detected by pathology) was cut from the isolated lung tissue during operation and fixed with 10% formaldehyde solution. Paraffin sections were prepared for AQP1 immunohistochemical staining, and AQP1-positive staining was observed under 100x, 200x, and 400x magnification under a light microscope, with brown-stained cells as positive expression cells. At 100x magnification, five positive visual fields were randomly selected from each slice, and the average integrated optical density (IOD) and average optical density (OD) of positive cells were calculated by using Image-Pro Plus 6 image analysis system.

#### 2.6.2. Detection of AQP1 Protein Expression Level

Six patients were randomly selected from the two groups. Normal lung tissues with the size of 1 × 1 × 1 cm^3^ (more than 5 cm away from tumor and nontumor tissues detected by pathology) were cut from the isolated lung tissues and stored in an 80 ultralow-temperature refrigerator, and the expression level of AQP1 protein was determined by Western blot. The gray value of the target protein was detected by Quantity One software, and the relative expression of target protein is equal to the target protein gray value/GAPDH gray value.

RETRACTED

### 2.7. Diagnostic Criteria of Postoperative Pulmonary Complications (PPCs) [12]

#### 2.7.1. Atelectasis

Atelectasis is found on chest CT or X-ray.

#### 2.7.2. Postoperative Pneumonia

(1) Postoperative pneumonia is diagnosed if at least two of the following are present: (a) new cough, dyspnea, or increased respiratory frequency or aggravation of original symptoms; (b) changes in the character of new purulent sputum or sputum, or an increase in respiratory secretions, or the need for sputum suction; (c) physical examination found lung rale or tubular breathing; (d) gas exchange worsened, oxygen demand increased, or ventilator-assisted breathing was needed. (2) Postoperative pneumonia is diagnosed if at least one of the following is present: (a) fever (*T* > 38.0°C) with no other explanation; (b) peripheral blood leukocyte count < 4 × 10^9^/L; or >12 × 10^9^/L for people older than 70 years old, there is an unexplained change in mental state. (3) Chest X-ray examination showed recent or progressive infiltration, consolidation, cavity, and pleural effusion.

#### 2.7.3. Acute Respiratory Distress Syndrome

(1) There are new respiratory symptoms or aggravation of original respiratory symptoms within 1 week. (2) For the chest image, chest radiograph or CT showed that the transmittance of both lungs decreased, which could not be completely explained by effusion, atelectasis, or nodules. (3) In pulmonary edema, respiratory failure cannot be explained by heart failure or excessive fluid load (objective evaluation, such as echocardiography, is needed to eliminate pulmonary edema caused by elevated hydrostatic pressure). (4) Under PEEP or CPAP ≥ 5 mmH_2_O ventilation, oxygenation index < 300 mmHg.

### 2.8. Statistical Analysis

The statistical method was analysed by SPSS 20.0 statistical software, and the measurement data were expressed by mean standard deviation ($\bar{x}\pm s$). Independent-sample *t*-test was used between groups, and repeated measurement variance analysis was used for comparison among multiple time points within groups. Counting data is expressed as percentage (rate), and chi-squared test is used for comparison; the abnormal distribution data were expressed by median and total distance, and Mann-Whitney *U* test was used for comparison between groups. The test level is *α* = 0.05, that is, *P* < 0.05 indicates that the difference is statistically significant.

RETRACTED

## 3. Results

### 3.1. General Conditions between Two Groups of Patients

There is no statistical difference in general data (age, sex, BMI, ASA grade, and surgical site) between the two groups (*P* > 0.05), as shown in Tables 1 and 2.

### 3.2. Comparison of Intraoperative Situations

There was no significant difference in operation time, blood loss, infusion volume, propofol dosage, and OLV time between the two groups (*P* > 0.05), as shown in Table 3.

### 3.3. Comparison of Intraoperative Center Rate (HR), Mean Arterial Pressure (MAP), Oxygenation Index (OI), and Alveolar Arterial Oxygen Partial Pressure Difference (A-aDO_2_)

There was no significant difference in HR and MAP between the two groups (*P* > 0.05). At T0, T1, and T2, there was no significant difference in OI and A-aDO_2_ between the two groups (*P* > 0.05). At T3, compared with group C, OI in group D increased and A-aDO_2_ decreased, with statistical difference (*P* < 0.05) (Table 4).

### 3.4. Comparison of the Incidence of Bradycardia and Hypotension in Operation Center between the Two Groups

Compared with the two groups during operation, the incidence of bradycardia in group D was higher and atropine was used more, with statistical difference (*P* < 0.05). There was no significant difference in ephedrine dosage (*P* > 0.05), as shown in Table 5.

### 3.5. Comparison of Serum IL-8 Concentration

At T0, there was no significant difference in serum IL-8 concentration between the two groups (*P* > 0.05). Compared with T0, the concentration of IL-8 in both groups increased significantly at T2 (*P* < 0.05). At T2, the concentration of IL-8 in group D was lower than that in group C (*P* < 0.05), as shown in Table 6 and Figure 1.

### 3.6. Comparison of Average Optical Density of AQP1

Immunohistochemical results showed that AQP1 was mainly distributed in pulmonary capillary endothelial cells and alveoli, and the average optical density of AQP1 in the lung tissue of the two groups was significantly different (*P* < 0.05). Compared with group C, the average optical density of group D was significantly higher, and the expression intensity of AQP1 in the lung tissue was significantly enhanced (*P* < 0.05), as shown in Figure 2 and Table 7.

### 3.7. The Expression of AQP1 Was Determined by Western Blot

Compared with group C, the gray value of AQP1 in group D was higher, and the color of the developing strip was wider and deeper, which showed that the expression of AQP1 in group D was higher (*P* < 0.05), as shown in Table 8 and Figure 3.

RETRACTED

### 3.8. Comparison of Postoperative Hospital Stay, Atelectasis, Pneumonia, ARDS, and Incidence of PPCs

There was no significant difference in postoperative hospital stay, atelectasis, pneumonia, ARDS, and PPC incidence between the two groups (*P* > 0.05). (Table 9).

## 4. Discussion

In clinical anesthesia for thoracic surgery, in order to provide a good surgical vision, one-lung ventilation technique is often used. This technique belongs to the nonphysiological breathing mode, which can easily cause acute lung injury (ALI). The inflammatory reaction of thoracic surgery is more serious than that of abdominal surgery. Hypoxemia caused by one-lung ventilation (OLV) during thoracic surgery leads to the increase of inflammatory factors [13, 14], and a large number of inflammatory mediators attack the lung tissue, resulting in lung injury. During one-lung ventilation, mechanical ventilation mode generally adopts volume control (VCV) or pressure control (PCV), and there is no significant difference in postoperative complications and prognosis between the two modes. Compared with PCV, VCV has the characteristics of higher platform pressure, higher volume, and less dead space ventilation. During operation, VCV can maintain higher arterial oxygen partial pressure and oxygenation index, but the peak airway pressure and inflammatory factor level are higher. For patients with poor lung compliance, the probability of lung injury is higher [11, 15]. In this experiment, we adopted the protective ventilation strategy and set the breathing parameters as follows: VT = 6 − 8 mL/kg, f = 12-15 times/min, PEEP = 5 cmH_2_O, *I*/*E* = 1 : 2, FIO_2_ = 1.0, and we adjusted the breathing frequency to keep PETCO_2_ in the range of 35-45 mmHg, so as to minimize air pressure injury. However, whether in animal experiments or human observation studies, it is found that “protective ventilation strategy” cannot completely prevent the massive production of inflammatory mediators in the lung and the subsequent damage to the lung tissue.

ALI is a pathological process characterized by increased permeability of the lung and inflammatory reaction of the lung. IL-8 stimulates chemotactic neutrophils to gather in the airway, alveoli, and other tissues, which promotes airway inflammation and aggravates it. Many studies have confirmed that IL-8 plays an important role in the pathogenesis of lung injury and pulmonary interstitial diseases, and its concentration reflects the degree of lung injury to a certain extent [16]. Aquaporins (AQPs) are a kind of cell membrane proteins related to the transmembrane transport of water and specifically transporting water. AQP1 is the first discovered AQP proteins, its molecular weight is 28 kDa, the gene locates on human chromosome 7p14, and its basic structure is a monomer composed of six transmembrane helical segments and two short helical segments without transmembrane. At the same time, every four AQP1 monomers form a stable tetramer on the cell membrane, and an independent water pore channel is formed in the middle [17]. AQP1 is mainly distributed in the lung tissue, with the strongest expression in pulmonary capillary endothelium and the weaker expression in alveolar cells. AQP1 can reflect the ability of clearing water in the lung tissue. Therefore, the concentration of IL-8 and the expression level of AQP1 were selected as detection indexes in this experiment.

RETRACTED

Dexmedetomidine, as a sedative drug widely used in clinical anesthesia, has the effect of inhibiting inflammatory reaction [18]. The commonly used clinical dose is intravenous pump loading of 1 *μ*g/kg and then continuous pump loading of 0.2-0.7 *μ*g/kg/h. In the experiment, patients in the dexmedetomidine group chose the usual dose of dexmedetomidine in clinical anesthesia. Dexmedetomidine inhibits the sympathetic nerve, and the incidence of intraoperative hypotension and bradycardia is high, which can be antagonized by atropine and ephedrine. There was no statistical difference in blood pressure and heart rate between the two groups, and it has no effect on the prognosis of patients.

There was no statistical difference between the two groups of thoracoscopic surgery cases. The results showed that at T2, the concentration of IL-8 in the two groups was significantly higher than that at T0 (*P* < 0.05), and the IL-8 in the two groups was significantly higher during operation than before operation. It showed that the inflammatory reaction of the body was obviously enhanced during operation and one-lung ventilation, which is difficult to avoid even by adopting lung protective ventilation strategy and dexmedetomidine. At the same time, thoracic surgical trauma and tumor itself (benign or malignant) could also cause inflammatory reaction [19, 20]. After the application of dexmedetomidine, the level of IL-8 in group D was significantly lower than that in group C, which indicated that dexmedetomidine could inhibit the production of IL-8, alleviate the inflammatory reaction, and protect the body. This result was consistent with many studies at present. There are many mechanisms for dexmedetomidine to inhibit inflammatory reaction, mainly because it acts on *α*-2 adrenergic receptor and reduces catecholamine secretion. When yohimbine (*α* receptor antagonist) was used, its inhibitory effect on inflammatory factors (tumor necrosis factor *α*, IL-6, and IL-8) could be reversed [21]. Other studies have found that it could inhibit inflammatory reaction through a variety of cellular pathways, which may be related to the downregulation of TLR4 expression in monocytes [22], which were the main source of IL-8 production.

RETRACTED

Immunohistochemical detection of AQP1 and Western blot were performed in the isolated lung tissues. Both methods confirmed that the expression of AQP1 in group D was significantly higher than that in group C (*P* < 0.05). In thoracic surgery, long-term one-lung ventilation can lead to increased permeability of pulmonary capillaries and increased vascular exudation, showing interstitial edema of the lung [23]. In the experiment, the expression of AQP1 in the dexmedetomidine group was enhanced, which can promote the flow of liquid inside and outside the cell membrane, enhance the body's ability to remove excessive edema liquid in the alveolar cavity and interstitial lung, improve the fluid balance in the lung, reduce the accumulation of water, prevent pulmonary edema, and improve the prognosis. Our results verified our scientific hypothesis that dexmedetomidine inhibited the production of IL-8 and promoted the expression of AQP1. However, due to the limitation of detection means, the specific process of regulation mechanism needs further study.

In the experiment, it was observed that there was no significant difference in OI and A-aDO_2_ between the two groups at T0, T1, and T2 (*P* > 0.05). At T3 (when the patient left the operating room to breathe air), the OI in the experimental group was higher than that in the control group, and the A-aDO_2_ was lower than that in the control group (*P* < 0.05). We believe that dexmedetomidine can improve the oxygenation and diffusion function of the lung, mainly because it inhibits the release of inflammatory factors and promotes the expression of AQP1. After dexmedetomidine was used, the production of IL-8 decreased, which could reduce the damage of alveolar epithelial cells and capillary endothelial cells in the alveoli, maintain the normal function of cell membrane, and promote the gas exchange in the lung. At the same time, the upregulation of AQP1 expression can accelerate fluid movement in the lung, reduce diffuse interstitial lung and alveolar edema, promote water balance in the lung, and improve hypoxia and diffusion function. In addition, the central channel of AQPs can directly pass through oxygen molecules, thus increasing the permeability of “gas-blood barrier” to oxygen, promoting oxygen transmembrane transport, and maintaining oxygen steady state, thus improving oxygenation function [24]. In addition, dexmedetomidine can also weaken the inhibitory effect of other anesthetics on hypoxic pulmonary vasoconstriction (HPV) and then improve the ratio of pulmonary ventilation to the blood flow [25]. By dilation of the bronchi, the dead space ventilation is reduced and the dynamic compliance of the lung is improved [26, 27]. It can also activate the *α*-2 receptor of vascular endothelial cells to release nitric oxide (NO), which can reduce vascular resistance in pulmonary ventilation area, reduce intrapulmonary shunt, and improve oxygenation [28].

RETRACTED

The incidence of pulmonary complications after thoracic surgery (14-59%) was much higher than that of upper abdominal surgery (16-17%) and lower abdominal surgery (0-5%) [29]. We counted the incidence of PPCs in patients, and there was no statistical difference between the two groups, which was not consistent with the hypothesis that dexmedetomidine suppressed inflammation and upregulated AQP1 expression could improve the prognosis. It was considered to be related to insufficient sample size and more clinical interference factors. The occurrence of PPCs was also affected by many independent risk factors, such as smoking, advanced age (≥75 years old), decreased mobility, ASA score ≥ 3, cardiovascular disease, COPD, and BMI > 30 kg/m^2^. Although the exclusion criteria were clearly defined in the experiment, all risk factors were balanced as far as possible, but clinical research will inevitably be affected by many factors. Lee et al. counted 50 cases of lung cancer and did not find that the incidence of PPCs decreased significantly after the administration of dexmedetomidine [25], but the number of statistical cases was also less. In the animal experiment, in the rats undergoing pneumoperitoneum operation, the alveolar structure of the lung tissue in the control group was seriously damaged, the alveolar septum was thickened, and a large number of leukocyte infiltration, edema, and diffuse hemorrhage could be seen. The incidence of leukocyte infiltration, edema, and hemorrhage was lower in the right medetomidine group [30]. Although the clinical study did not get the positive results of dexmedetomidine in improving postoperative pulmonary complications, from the animal experiment, the protective effect of dexmedetomidine on the lung was obvious to all. Therefore, combined with the experimental results of serum IL-8 and AQP1 expression, we believe that we cannot deny the hypothesis that dexmedetomidine can protect the lung by inhibiting the production of IL8 and upregulating the expression of AQP.

## 5. Conclusion

To sum up, we believe that the clinical dose of dexmedetomidine can inhibit the release of inflammatory factors, promote the expression of AQP1 in the lung tissue, and prevent lung injury.

RETRACTED

## Figures and Tables

**Figure 1:** Serum IL-8 concentration of two groups of patients. Compared with T0, ^#^*P* < 0.05; compared with group C, ^∗^*P* < 0.05.

**Figure 2:** Expression of AQP1 in the lung tissue. (a) alveolar and surrounding tissues in group C, ×200; (b) alveolar and surrounding tissues in group D, ×200; (c) alveoli and surrounding tissues in group C, ×400; (d) alveoli and surrounding tissues in group D, ×400.

**Figure 3:** Western blot detection of AQP1 expression in the isolated lung tissue. Control group: A, B, C, D, E, and F; group C: G, H, I, J, K, and L.

**Table 1:** Comparison of general data (*n* = 20).

Group	Age ($\bar{x}\pm s$, years)	Sex (*n*, male/female)	BMI ($\bar{x}\pm s$, kg/m^2^)	ASA stage (*n*, I/II)
Group C	58 ± 9	11/9	23.9 ± 3.3	6/14
Group D	52 ± 8	13/7	24.9 ± 3.5	8/12

**Table 2:** Comparison of surgical sites (cases (rate%)).

Group	Cases (*n*)	TL			
		Left upper lobe	Left lower lobe	Right upper lobe	Lower right lobe
Group C	20	4 (10)	5 (25)	6 (30)	5 (25)
Group D	20	5 (25)	4 (20)	4 (25)	7 (35)

**Table 3:** Comparison of intraoperative situations.

Group	Operation time (min)	Blood loss (mL)	Infusion volume (mL)	Propofol dosage (mg)	OLV time (min)
Group C	149.0 ± 37.9	85.3 ± 34.0	1155 ± 182	937.5 ± 183.4	124.5 ± 42.2
Group D	152.5 ± 47.7	88.8 ± 35.1	1170 ± 229	889.3 ± 192.3	126.0 ± 45.1

**Table 4:** Comparison of HR, MAP, OI, and A-aDO_2_.

Indicators	Groups	T0	T1	T2	T3
HR (times/min)	Group C	68.60 ± 9.82	63.70 ± 6.74	62.75 ± 5.99	66.25 ± 8.14
	Group D	69.15 ± 9.13	62.25 ± 4.33	61.80 ± 4.44	65.75 ± 7.93
MAP (mmHg)	Group C	96.45 ± 5.87	86.10 ± 4.56	85.00 ± 3.84	94.05 ± 5.16
	Group D	97.40 ± 6.99	84.95 ± 5.64	84.30 ± 6.15	93.55 ± 5.38
OI	Group C	371 ± 38	319 ± 52	105 ± 32^#^	312 ± 32^#^
	Group D	383 ± 34	340 ± 48	121 ± 28^#^	363 ± 34^#^^∗^
A-aDO_2_	Group C	9.75 ± 2.90	183.15 ± 54.73^#^	409.15 ± 39.54^#^	20.48 ± 6.35^#^
	Group D	9.45 ± 2.84	180.10 ± 53.80^#^	398.25 ± 40.39^#^	12.50 ± 4.37^∗^

^#^ *P* < 0.05 compared with T0; compared with group C, ^∗^*P* < 0.05. The local altitude was about 1880 meters.

**Table 5:** Comparison of incidence of intraoperative bradycardia and hypotension (*n* = 20).

Group	Bradycardia (cases (rate%))	Hypotension (cases (rate%))
Group C	2 (10)	1 (5)
Group D	8 (40)^∗^	7 (35)^∗^

^∗^Compared with group C, *P* < 0.05.

**Table 6:** Comparison of serum IL-8 concentration.

Group	T0	T2
Group C	213.72 ± 39.96	281.04 ± 54.59^#^
Group D	209.03 ± 39.62	244.38 ± 49.48^#^

Compared with T0, ^#^*P* < 0.05.

**Table 7:** Comparison of average optical density (*n* = 20 ($\bar{x}\pm s$).

Group	IOD	Average optical density
Group C	211140.70 ± 58234.68	0.52 ± 0.14
Group D	68178.60 ± 18188.17	0.94 ± 0.24
*t*	-10.48	6.69
*P*	<0.05	<0.05

RETRACTED

**Table 8:** Comparison of postoperative hospital stay, atelectasis, pneumonia, ARDS, and incidence of PPCs (*n* = 20).

Group	Postoperative hospital stay (d, $\bar{x}\pm s$)	Atelectasis (cases (%))	Pneumonia (cases (%))	ARDS (cases (%))	PPCs (cases (%))
Group C	4.60 ± 1.88	2 (10)	2 (10)	0 (0)	2 (10)
Group D	4.10 ± 1.48	1 (5)	2 (10)	0 (0)	2 (10)

**Table 9:** The expression of AQP1 protein (median (full distance)) (*n* = 20).

Group	AQP1
Group C	0.29 (0.14~0.39)
Group D	1.28 (0.22~1.77)^∗^

^∗^Compared with group C, *P* < 0.05.

## Data Availability

All the data could be provided if any qualified author required.
